This article has been retracted.

# Application of 3D Printing Technology and Porous Nano-Ceramic Decorative Sheet in Interior Landscape Design

**DOI:** 10.1155/2022/8715211

**Published:** 2022-11-08

**Authors:** Baojin Qiu, Xun Xu

**Affiliations:** School of Art, East China University of Technology, Nanchang 330032, Jiangxi, China

## Abstract

In order to solve the problems that the traditional ceramic method is difficult to form porous ceramics with complex structures, the mold production cycle is long, and the cost is high, the authors propose the application of 3D printing technology and porous nano-ceramic decorative sheet in interior landscape design. Based on the use of photocuring molding technology to make high-precision regular resin molds, optimize the low-viscosity, high-solid content alumina ceramic slurry required by the gel injection molding process and form alumina ceramic blanks by means of a vacuum pressure process, so as to realize the net shape of complex structural porous ceramic parts. In view of the filling problem of ceramic slurry in complex structure in the process, the effects of slurry pH value, dispersant dosage, and vacuum pressurization process on ceramic molding were studied, and parameters such as porosity and compressive strength of the green body were tested. Experimental results show the following. Under the conditions of pH value of 9, mass fraction of dispersant of 0.4%, and vacuum pressure of 90 min, alumina ceramics with a volume fraction of 52% can be prepared, the porosity is 51.5%, and the compressive strength is 40.1 MPa. The ceramic material prepared by this process has complete structure and smooth surface and can be used as a process for preparing porous ceramic parts with complex structure.

## 1. Introduction

With the development and changes of the times, people's living environment has also undergone earth-shaking changes; because of the popularity of industrialization and the high-density gathering of people, people's living environment has developed from idyllic villages and small towns to cities with high-rise buildings [1]. The appearance of a large number of high-rise buildings makes people living in cities far away from nature, and green plants can rarely be seen in cities [2]. Therefore, in the current urban life, people have a higher desire for natural scenery, landscapes such as plants, rivers, and rocks can greatly relax the nervous nerves of urban people and improve people's mental state [3]. Due to this demand, people are constantly trying to migrate natural scenery indoors, which is also the origin of indoor landscape design.

The development of interior landscape design has mainly gone through three stages of modernism, post-modernism, and new modernism; with the emergence of the environmental crisis and energy crisis in the new era, the interior landscape design has gradually developed towards functionality and rationality, and the protection of the ecological environment has been the main goal [4]. Compared with the West, China's interior landscape design does not have the complicated and rich artistic genres of the West, but it also has its own unique artistic style and many years of successful experience. In China, people prefer the water bureau to set the scene. Besides, stone sets, plant sets, pavilions, and other styles of garden architecture are also Chinese people's preference. Through the combination of these elements, the interior can be formed into a very regional characteristics of the landscape, and in line with the aesthetic of Chinese people [5]. With the development and progress of the times, people's aesthetics and design requirements are improved, and interior landscape design is no longer limited to aesthetics and comfort but also requires interactivity and intelligence [6].

The technological innovations of the twenty-first century are largely underpinned by the understanding of more microscopic phenomena and the development of operational techniques accordingly. However, from a macro-perspective, the traditional technology development of pursuing a more micro-world will reach its limit in many fields. It is impossible to reach new heights without new discoveries that are fundamentally different from traditional techniques [7]. Nano-ceramic materials developed by nanotechnology refer to the microstructure of ceramic materials; the grains, grain boundaries, and the combination between them are all at the nanometer level (1–100 nm), which greatly improves the strength, toughness, and superplasticity of the material; it overcomes many shortcomings of engineering ceramics and has an important impact on the mechanical, electrical, thermal, magnetic, optical, and other properties of materials, and it has opened up a new field for the application of alternative engineering ceramics [8]. With the wide application of nanotechnology, nano-ceramics are produced, hoping to overcome the brittleness of ceramic materials and make ceramics as flexible and machinable as metals. Nanometer high temperature resistant ceramic powder coating material is a material that forms a high temperature resistant ceramic coating through chemical reaction [9].

## 2. Literature Review

The application of ceramics has a long history in our country. From traditional ceramics used in daily life to modern electronic ceramics, structural ceramics, and other special ceramics, the application scope of ceramics has undergone great changes; because of its high temperature resistance, high hardness, and high thermal conductivity, it has attracted much attention from scholars [10]. The traditional method of preparing ceramics is to mix, shape, and sinter various raw material powders to obtain ceramic parts. However, due to the high temperature required for ceramic sintering, the shape, size, and properties are easily affected by the sintering process, and the ceramic itself is brittle and difficult to reprocess after sintering; therefore, some ceramics with high surface quality and precision are difficult to obtain by traditional preparation techniques [11]. 3D printing technology plays an important role in solving this problem.

According to the model in the document, the 3D laser printing technology uses the adhesive material from the bottom layer to print layer by layer, and then combines into the 3D object model [12]. With the continuous development of 3D laser printing technology, rapid prototyping technology has also made great breakthroughs and is widely used in many fields. Before traditional 3D printing, it is necessary to use related software to manually operate the virtual model, and the workload is large, time-consuming, and laborious, which greatly increases the difficulty of reconstruction; at the same time, the efficiency of the whole process from model design to 3D printing is reduced [13].

Porous ceramic materials are different from traditional ceramic materials because of the many pores in their structure; they have the characteristics of low apparent density, light relative weight, sound absorption and heat insulation, and good filterability and adsorption, and they can be used in fluid separation and filtration, noise reduction, energy absorption and buffering, shielding electromagnetic signals, thermal insulation, heat exchange, and catalysts [14]. Due to the poor conductivity, high hardness, and high melting point of ceramics, many complex shapes of high-strength and high-performance ceramic structural parts are difficult to directly form. Gel injection molding technology can not only obtain green embryos with high mechanical strength, but also not limited by complex molding shapes and sizes, but the limitation of mold dependence makes the product design cycle longer [15]. Gel injection molding technology can not only obtain high mechanical strength embryo but also be free from complicated shape and size. However, the limitation of dependence on the mold makes the product design cycle longer. This method can not only easily obtain porous ceramic materials but also change the shape of the mold at any time as needed, which is conducive to various comparisons and experiments and requires less equipment and raw materials, and the process is simple; it provides a reference for the preparation of porous ceramic parts with complex structures [16]. There are two main factors that affect the structural integrity of ceramic slurry in the process of filling complex structural molds: one is the rheology and stability of the ceramic slurry itself; the other is that in the general mold filling process, the ceramic slurry can be completed only by the gravity of the slurry itself; however, for complex structure molds, it is difficult to meet the filling requirements in microstructures only by the action of gravity [17]. The research group mainly takes these two points as the research content: Alumina ceramic slurry with good uniformity, fluidity, stability, and high solid content will be prepared;The filling requirement of ceramic paste in complex structure will be realized by using the driving force given by vacuum pressure device.

## 3. Methods

### 3.1. Analysis of Mechanical Properties of Ceramic Materials

In the case of impact and compression loading of ceramics, the microcrack surface of ceramic materials at the mesoscopic level leads to discontinuous deformation or displacement discontinuity, and at the same time, it also leads to the collapse of pores [18]. Assuming that *ℰv* represents the state variable on the destruction front, its governing equation can be expressed as follows:

(1) $$\begin{array}{c} f\left(x\right)=\left(\frac{\varepsilon v}{t}+C_{F}\frac{\varepsilon v}{X}\right)\times \xi \left(X,t\right)\text{,} \end{array}$$

where *t* represents the transportation time, *C*_*F*_ represents the propagation velocity of the failure wave, and *X* represents the surface area of the microcrack; then, the value range of the pore collapse area function *ξ*(*X*, *t*) is as follows:

(2) $$\begin{array}{c} \xi \left(X,t\right)=\frac{\tau C_{0}}{\tau_{HEL}}H\left(\tau -\tau_{THD}\right)\text{,} \end{array}$$

where *C*_0_ represents the material parameter; H represents the Heaviside function; *τ*_THD_ represents the shear stress threshold of the microcrack system formed by the ceramic under shock compression; and *τ*_HEL_ represents the macroscopic shear stress when the material reaches the limit state, which corresponds to the transition of the microcrack system in the ceramic material [19]. For fragile materials, since hydrostatic pressure and shear stress jointly affect the inelastic deformation and failure response of the material, the value range of the fragility function *τ*(*X*, *t*) of the ceramic material is

(3) $$\begin{array}{c} \tau =\frac{\sqrt{3}}{2}\Phi \left(I_{1}+\sqrt{J_{2}}\right)\text{.} \end{array}$$

Among them, the hydrostatic pressure *I*_1_ and shear stress *J*_2_ are, respectively, expressed as

(4) $$\begin{array}{c} I_{1}=\gamma_{ij}\text{,} \end{array}$$

(5) $$\begin{array}{c} J_{2}=0.5\gamma_{ij}^{2}\text{,} \end{array}$$

where Φ represents the failure wave parameter and *γ*_*ij*_ represents the material parameter, and the value of the parameter *γ*_*ij*_ mainly depends on the microstructure of the material. For glass materials, when the impact compressive strength reaches the set range, the formation of damage waves can be observed [20]. If Φ=0.5 is set, under the condition of one-dimensional strain, the above formula can be degenerated into

(6) $$\begin{array}{c} \tau =\frac{1}{2}\Phi \left[\sqrt{3}\left(\sigma_{1}+2\sigma_{2}\right)+\left|\sigma_{1}-\sigma_{2}\right|\right]\text{,} \end{array}$$

where *σ*_1_ represents the longitudinal stress and *σ*_2_ represents the transverse stress.

For the propagation of the destructive wave, it is assumed that the destructive wave front is located at position *A* at time *t* and reaches position *B* after *d*_*t*_ time period. The specific expression formula of the mechanical energy conservation equation is given below:

(7) $$\begin{array}{c} G=C_{F}W+C_{F}\left(\sigma -vd_{t}\right)+\frac{1}{2}J_{2}D\text{.} \end{array}$$

The mechanical energy flux density can be expressed as

(8) $$\begin{array}{c} W=-\left[\sigma *v\right]*n\text{.} \end{array}$$

The mechanical energy dissipation rate is

(9) $$\begin{array}{c} D=\frac{\xi \left(X,t\right)}{\tau }+\varepsilon v\text{.} \end{array}$$

For fragile materials, the inelastic expansion volume strain *EcV* is mainly caused by the expansion of microcracks; combined with relevant theories, one-dimensional strain compression can be obtained, and then there is

(10) $$\begin{array}{c} d\varepsilon_{V}^{e}=d_{t}\cdot \frac{1}{3-\tan\;\varphi }\left[\sqrt{\frac{3}{J_{2}}\left(\sigma_{1}-\sigma_{2}\right)+\tan\;\varphi }\right]\text{.} \end{array}$$

When the stress state in the material under shock compression needs to meet the corresponding failure criterion, the nucleation and expansion of microcracks in the material mainly transition along the microcrystalline crack to the transgranular crack, and the relationship between the porosity of the material and the hydrostatic pressure can be expressed in the following form:

(11) $$\begin{array}{c} n=n_{HEL}-C_{c}\frac{H}{\tau_{HEL}}\text{,} \end{array}$$

where *n*_HEL_ represents the porosity of the material when the hydrostatic pressure is *p*_HEL_ and *C*_*c*_ stands for compression factor. The relationship between shock compressive stress, failure volume, and initial porosity is given below:

(12) $$\begin{array}{c} n_{HEL}=\frac{I_{1}\cdot f\left(x\right)}{C_{c}}\text{.} \end{array}$$

In order to accurately describe the variation law of transverse pressure under one-dimensional strain conditions, the failure factor of the material after failure filtering can be expressed as

(13) $$\begin{array}{c} K=\frac{G-C_{F}\times Ev}{n_{HEL}}\text{.} \end{array}$$

Combining the above formula, it can be seen that the failure factor of the material tends to the limit value 1 with the increase of the loading strength, and the relationship between Poisson's ratio *K* of the failure layer material and the failure factor *p* can be expressed as

(14) $$\begin{array}{c} K=\left(\frac{1}{2}\sigma_{1}-\sigma_{2}\right)\times p\text{.} \end{array}$$

Among them, the transverse stress under one-dimensional strain conditions can be expressed as

(15) $$\begin{array}{c} \sigma_{2}=\left\{\begin{array}{c} p\text{,}\\ \frac{1}{1-p}\sigma^{1} \end{array}\right.\text{.} \end{array}$$

### 3.2. Experiment

#### 3.2.1. Experimental Materials

The raw materials used in the experiment are alumina powder (average particle size is 200 nm), organic monomer methacrylamide (MAM), crosslinking agent methylenebisacrylamide (MBAM), catalyst tetramethylethylenediamine (TEMED), initiator ammonium persulfate (APS), dispersant DolapixCE64 (main component is polyammonium methacrylate), and ammonia. The equipment used in other experiments included light-curing 3D printers, casting resins, planetary ball mills, vacuum pressurizing devices, drying ovens, and tubular sintering furnaces, as shown in Table 1.

#### 3.2.2. Experimental Steps

The process flow of gel injection molding is shown in Figure 1. The process steps are as follows. ① Add alumina powder, organic monomer, crosslinking agent, and dispersant to solvent deionized water in a certain proportion, and it is mixed with a ball mill for a certain period of time to form a powder suspension slurry. ② Add initiator and catalyst before injection molding, and after fully stirring, inject the slurry into the mold and vacuumize/pressurize. ③ Under certain temperature conditions, the organic monomers are induced to undergo a gel reaction, so that the ceramic slurry is solidified and formed to form a green body with a certain strength. ④ Dry it at a certain temperature to obtain a green body with higher strength. ⑤ Demold simultaneously during the green body debinding and sintering process to obtain dense ceramic parts.

### 3.3. Analysis and Determination

Use MIK-pH meter to measure the pH value of the slurry; SNB-1A-J digital rotational viscometer to measure the viscosity of the slurry; Archimedes drainage method to measure the porosity of the ceramic material; and WES-100 universal testing machine to measure the green body compressive strength.

## 4. Results and Discussion

The ceramic particles in the slurry tend to settle under the action of gravity, and the stability of the slurry can be reflected by the degree of sedimentation. Slurry with a volume fraction of 50% was prepared separately, and a dispersant (PMAA-NH4) with a mass fraction of 0.2% was added, and the pH value was adjusted to different pH values with ammonia water; after thorough mixing, the sedimentation degree and viscosity of the slurry were measured.

The relationship between the sedimentation rate and pH value is shown in Figure 2. As can be seen from the figure, when the pH value is around 9, the degree of sedimentation is small, indicating that the slurry stability is better at this time. The relationship between slurry viscosity and pH value is shown in Figure 3. With the increase of pH value, the viscosity of the slurry gradually decreased and reached the lowest at pH value of 8.5. With the increase of pH value, the viscosity of the slurry showed an upward trend.

On the one hand, the dispersant will dissociate in the slurry to generate acid ions and NH_4_^+^ ions; when the pH value is small, the dissociation degree *α* of the dispersant is also small, and the polymer electrolyte is easy to agglomerate, resulting in a decrease in the dispersibility of the slurry. When the pH value is high, the degree of dissociation *α* also increases; under the action of static electricity, the alumina particles will adsorb more acid ions, which will increase the negative charge on the surface, thereby increasing the electrostatic repulsion. On the other hand, according to colloid theory, when the ceramic slurry is alkaline as a whole, the surface charge of the particles is large, the zeta potential increases, the electrostatic repulsion between the particles is enhanced, the van der Waals force is small, the electrostatic force between particles is the strongest, and the slurry is in a relatively stable state; at this time, the absorption of acid ions by alumina particles reaches saturation. After continuing to increase the pH value, the excess polymer electrolyte in the slurry system will increase the viscosity of the slurry; therefore, when the pH value is alkaline (about 8.5 to 10.0), the dispersion stability of the slurry is the best.

The slurries with a volume fraction of 50% were prepared, respectively, the pH value was adjusted to 9 with ammonia water, and dispersants (PMAA-NH4) with different mass fractions were added, respectively, and the sedimentation degree and viscosity of the thin slurry were measured after thorough mixing.

The relationship between the sedimentation rate and the mass fraction of dispersant is shown in Figure 4. With the increase of the mass fraction of dispersant, the sedimentation rate of the slurry showed a downward trend; when the mass fraction of the dispersant was 0.3%, the sedimentation rate of the slurry reached the minimum. After continuing to increase the dispersant, the slurry settling rate increased slightly. The relationship between the viscosity of the slurry and the mass fraction of the added dispersant is shown in Figure 5. As the mass fraction of dispersant increases, the viscosity of the slurry also decreases, and when the mass fraction is 0.4%, the viscosity of the slurry reaches the minimum. The mass fraction continued to increase, and the viscosity of the slurry also increased.

From the point of view of double layer effect, the anion formed by adsorbing dispersant on the surface of alumina particles is dissociated. Anions adsorb part of the anti-charge ions in the solvent medium by electrostatic action, forming a whole with a double electric layer. It is negatively charged and stabilized by the repulsion of same charges. From the perspective of steric hindrance effect, the polymer dispersant has two kinds of groups: insoluble and soluble, in which the insoluble group will be attached to the surface of alumina particles, the soluble group is fully extended in the solvent medium, and the two make the spatial position of the particle in the solvent medium more stable; reducing the sedimentation of alumina particles also makes the surface of the particles more wet, reducing the friction between particles to reduce the viscosity. If the mass fraction of counter ions is increased in the solvent medium, that is, the mass fraction of dispersant is increased, the remaining counter ions will be forced into the counter ion layer on the particle surface due to electrostatic repulsion; in this way, the charge repulsion of the electric double layer is reduced, and the whole system tends to agglomerate and become unstable. Therefore, the research group selected a dispersant mass fraction of 0.4%.

Due to the gel injection molding process, air will inevitably be mixed in the process of ball milling, slurry preparation, and injection molding, forming pores, resulting in uneven internal density of the green body, affecting the strength, elastic modulus, and thermal conductivity of ceramic materials. The use of vacuuming process after injection molding can effectively discharge the air in the slurry and reduce the porosity. The main function of the pressurization process is to increase the filling power of the ceramic slurry, so that it can complete the flow in the complex and small structure and improve the filling ability of the ceramic slurry.

The alumina slurry was prepared with a volume fraction of 52%, a pH value of 9, and a mass fraction of dispersant of 0.4%, and it can be seen that the surface of the green body obtained by vacuum pressing for 90 min is smooth and clean, and the molding effect is good. On the one hand, if the pressure is too large, the ceramic slurry will have a certain degree of elastic deformation; when the pressure is released, the ceramic body will undergo a certain volume deformation. On the other hand, if the time is too long, the process will be lengthy, so the effect of the blank after 90 minutes of vacuum pressure is enough to meet the needs of filling.

Under the condition of vacuum pressure for 90 min, the volume fraction of alumina ceramic slurry was 52%, the pH value was 9, the mass fraction of dispersant was 0.4%, the ceramic materials was produced. Alumina ceramic parts were obtained after the degrease-stripping process in tube furnace 600°C and sintering of 1650°C for 2 hours. The porosity of the green body is 51.5% measured by the Archimedes method. The compressive strength is 44.1 MPa. The sample is relatively flat as a whole and has micron-scale pores, which can be used in catalyst carriers and filter materials.

## 5. Conclusion

The authors propose the application of 3D printing technology and porous nano-ceramic decorative sheet in interior landscape design; from a series of new and high properties such as ductility and superplasticity exhibited by nano-ceramics, it fully presents potential broad application prospects, but most preparation technologies are still in the experimental research stage, and only a few have entered the application stage; moreover, there are problems such as low output, high cost, and difficulty in industrial production, and the collection and storage of nano-powders are also difficult. The research and development of nano-ceramics will inevitably lead to the development and reform of the ceramic industry, as well as the development of ceramic theory and even the establishment of a new theoretical system, in order to meet the needs of nano-scale research; the nano-ceramic materials have better properties, so the emergence of new properties and functions is possible. We look forward to the wider application of nano-ceramics in engineering fields and even in daily life.

## Figures and Tables

**Figure 1:** Gel injection molding process flow.

**Figure 2:** Relationship between sedimentation rate and pH value.

**Figure 3:** Relationship between viscosity and pH value.

**Figure 4:** Relationship between sedimentation rate and mass fraction of dispersant.

**Figure 5:** Relationship between viscosity and mass fraction of dispersant.

**Table 1:** Experimental materials and equipment used.

Experimental raw materials	Experiment equipment
Alumina powder (average particle size is 200 nm)	Light-curing 3D printer
Organic monomer methacrylamide (MAM)	Casting resin
Crosslinker methylenebisacrylamide (MBAM)	Planetary ball mill
Catalyst tetramethylethylenediamine (TEMED)	Vacuum pressurizing device
Ammonium persulfate (APS)	Drying oven
Ammonium polymethacrylate ammonia	Tube sintering furnace

## Data Availability

The data used to support the findings of this study are available from the corresponding author upon request.
